The article "Measurement of Body Surface Area for Psoriasis Using U-net Models" was published in 2022. Journal: Comput Math Methods Med.

# Measurement of Body Surface Area for Psoriasis Using U-net Models

**DOI:** 10.1155/2022/7960151

**Published:** 2022-02-10

**Authors:** Yih-Lon Lin, Adam Huang, Chung-Yi Yang, Wen-Yu Chang

**Affiliations:** ^1^Department of Computer Science and Information Engineering, National Yunlin University of Science and Technology, Yunlin 64002, Taiwan; ^2^Department of Biomedical Sciences and Engineering, National Central University, Taoyuan City 32001, Taiwan; ^3^School of Medicine, College of Medicine, I-Shou University, Kaohsiung City 82445, Taiwan; ^4^Division of General Radiology, Department of Medical Imaging, E-Da Hospital, Kaohsiung City 82445, Taiwan; ^5^School of Medicine for International Students, College of Medicine, I-Shou University, Kaohsiung City 82445, Taiwan; ^6^Department of Dermatology, E-Da Cancer Hospital, Kaohsiung City 82445, Taiwan

## Abstract

During the evaluation of body surface area (BSA), precise measurement of psoriasis is crucial for assessing disease severity and modulating treatment strategies. Physicians usually evaluate patients subjectively through direct visual evaluation. However, judgment based on the naked eye is not reliable. This study is aimed at evaluating the use of machine learning methods, specifically U-net models, and developing an artificial neural network prediction model for automated psoriasis lesion segmentation and BSA measurement. The segmentation of psoriasis lesions using deep learning is adopted to measure the BSA of psoriasis so that the severity can be evaluated automatically in patients. An automated psoriasis lesion segmentation method based on the U-net architecture was used with a focus on high-resolution images and estimation of the BSA. The proposed method trained the model with the same patch size of 512 × 512 and predicted testing images with different patch sizes. We collected 255 high-resolution psoriasis images representing large anatomical sites, such as the trunk and extremities. The average residual of the ground truth image and the predicted image was approximately 0.033. The interclass correlation coefficient between the U-net and dermatologist's segmentations measured in the ratio of affected psoriasis over the body area in the test dataset was 0.966 (95% CI: 0.981–0.937), indicating strong agreement. Herein, the proposed U-net model achieved dermatologist-level performance in estimating the involved BSA for psoriasis.

## 1. Introduction

Psoriasis is a chronic immune-mediated skin disease with a global prevalence rate of approximately 2% [1]. It is a life-long, metabolic, immunological disorder characterized by raised areas of abnormal skin that wax and wane in the long-term course. The body surface area (BSA) of involvement is an important indicator during the evaluation of psoriasis severity. There are several treatment modalities, including topical medications, systemic immunomodulators, and phototherapies. Precise measurement of the affected BSA is important for clinicians to evaluate the treatment response when switching or combining these treatment options. It is also important for the clinical-trial investigators to monitor psoriasis severity when developing new therapeutic strategies [2]. Physicians usually evaluate the patient subjectively through direct visual evaluation, specifically the most widely used psoriasis area and severity index (PASI), and a recent tool, a product of the physician global assessment and BSA (PGA × BSA), which has the advantages of being more intuitive and easier to use than PASI. BSA is a crucial factor in the calculation of both methods when evaluating disease severity [3, 4]. Previous studies reported a high degree of variability during evaluation, and multiple interventional educational programs need to be conducted before starting the evaluation to achieve better accuracy and reliability [5, 6]. The increase of affected BSA also revealed the increasing burdens of overall medical and specific comorbid diseases, including cardiovascular, cerebrovascular, and diabetes risks [7, 8]. However, despite being such an important indicator, the affected BSA judgments are primarily based on the naked eye and previous physician impressions, which are both subjective and time-consuming.

There are different automatic segmentation methods for psoriasis lesions in the literature [9–16]. These include neuro-fuzzy classifiers [9, 10], *K*-means [11, 12], Gaussian mixture models [13], geometric active contours [14], support vector machines [15], and traditional shallow neural networks [16]. More recently, deeper neural network structures such as U-net have also been proposed to automate the segmentation of skin lesions in psoriasis images [17]. U-net was originally developed for biomedical image segmentation [18]. It is a relatively new technology based on a fully convolutional network [19] that can classify each pixel in an image into a specific label. Since its publication in 2015, it has quickly become one of the most popular tools for image segmentation with more than 24000 citations. Its success can be attributed primarily to its multiresolution structure encoder-decoder design, which can capture both large- and small-scale features for generating optimal segmentation results even with small training datasets [18]. Recently, researchers examined the U-net architecture and various developments and provided observations on recent trends [20].

In these studies, the authors chose the training and testing sets based on the same patch sizes with limited small fields [21–23]. However, test images from each patient are usually captured using various scales for clinical applications. In this study, the U-net model is adopted to develop an efficient way to estimate the psoriasis-to-total skin ratio by estimating the relevant BSA using the proposed methods.

## 2. Materials and Methods

### 2.1. Patient Collection

Adult patients over 20 years of age were recruited in this study, with a definite diagnosis of moderate-to-severe plaque-type psoriasis for over six months, and were candidates for phototherapy or systemic psoriasis treatment. The images were collected during follow-up schedules of psoriasis treatments according to the medical guidelines of the National Health Insurance of Taiwan. Photographs were obtained using a 22-megapixel digital single-lens reflex camera (5D Mark II, Canon Corporation, Tokyo, Japan) with 100 mm F2.8L microlens (Canon Corporation, Tokyo, Japan).

The ambient light was provided by two studio floodlights, D-Lite RX 4/4 softbox to go (Elinchrom SA, Renens, Switzerland) diffused by soft boxes positioned on both camera sides at 45° angles to the patient, and lights were positioned 1 m in front of the patient with a voltage of 5.5 V. A fixed distance of 2 m between the patient and the camera ensured standard reproduction ratios for whole-body imaging to monitor psoriasis treatment outcomes.

All patients provided written consent for image use, under privacy considerations. We separated facial images from others and excluded all facial images in this study. A dermatologist (W-Y C, with 16 years of experience) carefully reviewed the images and marked the psoriasis lesion border as the gold standard.

### 2.2. U-net Architecture

The U-net architecture for the segmentation of psoriasis skin lesions is illustrated in Figure 1. Based on the original U-net topology, it consists of the contraction path (or encoding path) and expansion path (or decoding path). The proposed architecture uses 24 convolutional layers, four max-pooling operations, four upsampling operations, and four concatenations. The contraction path uses eight convolution layers in conjunction with batch normalization and the ReLU activation function, followed by max-pooling. The max-pooling operation is performed after every two convolution operations. In the expansion path, upsampling is followed by 3 × 3 padded convolution, batch normalization, and activation layers, implemented sequentially to achieve better segmentation outcomes. A detailed explanation of each layer is provided in Table 1. The number of trainable weights in the proposed U-net is 31,035,971. Notably, “Cat-1” concatenates Conv-11 and Conv-8, “Cat-2” concatenates Conv-14 and Conv-6, “Cat-3” concatenates Conv-17 and Conv-4, and “Cat-4” concatenates Conv-20 and Conv-2.

Notably, in the U-net architecture, the convolution operation from the encoder and the deconvolution operation from the decoder are independent of both the input and output image sizes. In the testing process, the test image does not have to be resized to the size of the training image. Therefore, the model can be trained using one patch size and predict testing images of different sizes.

The performance of the proposed method was evaluated using five different indices, that is, accuracy (ACC), Dice coefficient (DSC), Jaccard index (JI), sensitivity (SE), and specificity (SP), in comparison with the ground truth. The overall pixel accuracy was measured for the skin, psoriasis, and background regions. The formulas for the performance indices are as follows:

(1) $$\begin{array}{c} \text{ACC}=\frac{\text{TP}+\text{TN}}{\text{TP}+\text{TN}+\text{FP}+\text{FN}}, \end{array}$$

(2) $$\begin{array}{c} \text{DSC}=\frac{2\text{TP}}{2\text{TP}+\text{FN}+\text{FP}}, \end{array}$$

(3) $$\begin{array}{c} \text{JI}=\frac{\text{TP}}{\text{TP}+\text{FP}+\text{FN}}, \end{array}$$

(4) $$\begin{array}{c} \text{SE}=\frac{\text{TP}}{\text{TP}+\text{FN}}, \end{array}$$

(5) $$\begin{array}{c} \text{SP}=\frac{\text{TP}}{\text{TN}+\text{FP}}, \end{array}$$

where TP denotes the true positives, FN denotes the false negatives, FP denotes the false positives, and TN denotes the true negatives.

In the experiments, we used 255 images of psoriasis lesions collected from 16 psoriasis patients, nine for training and seven for testing, by a dermatologist for various scales and working distances. Each image represents an anatomical site, and the final dataset includes 170 images of the extremities and 85 images of the truncal area (Table 2). The largest and smallest image sizes are 3744 × 5616 and 2017 × 1913, respectively. In our experiments, we first partitioned the dataset into training, validation, and testing datasets. The testing dataset consisted of newly collected data.

In our experiments, all training and validation images consisted of nonoverlapping patches of size 512 × 512. In other words, the size and stride of all extracted patches were 512 × 512 and 512, respectively. In these patches, there was an unequal distribution of skin, psoriasis, and background. To avoid the imbalance problem, we removed more background-only patches (i.e., the background patches containing no skin and psoriasis regions) using manual visualization from 9456 training and 2912 validation patches. The remaining 7809 training patches were used to train the model that included images of different body parts and quality, while the remaining 2048 validating images were used to validate the trained model. We wish to point out that we retained 49 testing images in their original sizes. The details are presented in Table 3.

## 3. Experimental Results

This section simulates and verifies the psoriasis estimation of the full-body surface using the proposed methods and the U-net model. Deep networks usually require a large amount of training data to achieve good performance. Data augmentation is a domain-specific technique that artificially creates new training data from preexisting training data. Our experiments used data augmentation with normalization, vertical and horizontal flips. The trajectories of the loss and accuracy for the training and validating data are shown in Figure 2. To evaluate the performance of the trained model, we used five performance indices defined in Equations (1)–(5) in comparison with the ground truth. The accuracy was measured for the skin, psoriasis, and background regions, while the remaining four indices were concerned only with psoriasis. To explain the performance more clearly, the resulting experimental images in both large scale (zoom out) and small scale (zoom in) are shown.

The summary statistics of the experimental results are listed in Table 4. In our experiments, we used 49 test images. However, to avoid division by zero in the calculation of the JI and DSC indices, we included 47 testing images for analysis. The mean and standard deviation of accuracy was 0.976 ± 0.046. The JI, DSC, SE, and SP of segmentation of psoriasis lesions were 0.536, 0.655, 0.657, and 0.988, respectively. The main reason for misclassification when segmenting the psoriasis area may be related to the small area of the diseased skin in general. By contrast, the high specificity could be attributed to the large areas of the skin and background.

Table 5 shows the values of the different metrics for the image with the lowest residual percentage. The accuracies of the large and small scales were 0.997 and 0.969, respectively. The values of JI, DSC, SE, and SP are listed from the third to the sixth columns. The images with the smallest residual percentage at different scales are shown in Figure 3. Figure 3 depicts the predicted image of psoriasis segmentation on a large scale for the lowest residual percentage, with the image inside the blue bounding box representing the small-scale image.

Images with the three largest residual percentages are shown in Figure 4. The figure clearly shows that the psoriasis area and severity are high. We could find severe psoriasis cases of patients in the testing image dataset but not in the training image dataset. Consequently, misclassifications can easily occur. Hence, it is advisable to collect more severe psoriasis data.

The distribution of the residual percentage of the psoriasis area estimation is shown in Figure 5. The five largest residual percentages are shown with green arrows, and the top three are shown with green dots. The lowest residual percentage is indicated in red. Statistics of the residual percentages for all the test images are listed in Table 6.

The ICC (two-way mixed model for absolute agreement, single measurement) was performed to conduct correlation agreement analysis for the U-net model versus dermatologist's manual segmentation for a test dataset of 49 images.  Figure 6 shows the resultant correlation scatterplots for U-net and dermatologist's segmentations measured in the ratio of affected psoriasis over the body area. The ICC of the test dataset was 0.966 (95% CI: 0.981-0.937). The concordance between the two estimation methods showed an excellent agreement (>0.90).  Figure 6 shows that when the psoriasis area extends over 40% of the body surface, most of the data points are above the line of agreement, demonstrating that the dermatologist segmented a larger psoriasis area at the high end of the scale than the U-net model.

The magnitude of agreement between U-net and dermatologist's measures was further quantified using Bland-Altman plots using all 49 test images.  Figure 7(a) shows that with all 49 test images, an average difference of -0.0266 (95% CI: 0.1283-0.1816, mean ± 1.96 SD) indicates a noticeable estimated bias, and the large bounds of the 95% confidence interval are caused by the reduced agreement for large body surface measurements. As the percentage of BSA increased, more estimation data of the U-net model fell below the expected 95% lower bound of agreement. By excluding the images with high psoriasis surface ratio and using only the psoriasis surface ratio lower than 50% to construct Bland-Altman plots, the average difference was improved to -0.00084 (95% CI: 0.0198–0.0215) (Figure 7(b)).

To provide a comparative analysis with the most recent approaches, apart from the proposed method, we used R2U-net [24], attention U-net [25], and attention R2U-net [26] for the problem under study.  Table 7 shows the number of parameters and file sizes for each learning model. For a more reasonable comparison, the learning models were configured such that their numbers of adjustable filters were approximately the same. The performances of the testing datasets for the proposed U-net, R2U-net, attention U-net, and attention R2U-net models are listed in Tables 8 and 9. The proposed model performs slightly better than the other three learning models. From a practical application viewpoint, all four learning models listed in Table 7 perform equally well, but the number of parameters in our proposed model is the smallest, which is usually desirable for practical implementation of the learning model, particularly on edge computing devices.

## 4. Discussion

This study makes several main contributions to the literature. In previous studies, most training and testing images were cropped into many small-scale patches with a few papules or plaques [17, 21, 22]. In our research, all testing images were captured using a digital camera under the medical practice guidelines. The proposed U-net model was used to estimate large-scale images of anatomical regions rather than a few focal lesions. This contributes to the applicability of direct and massive use in future clinical studies.

We selected the U-net model because of its popularity and easy accessibility. This study demonstrated that the JI and DSC of this model performed moderately. However, the U-net model-generated segmentation shows excellent agreement with the dermatologist-generated manual segmentation for estimating the BSA percentage, supporting the applicability of the tool for clinical use. We observed that the U-net model tends to underestimate 11 severe cases with psoriasis areas larger than 40%. The margins of psoriasis are not always clear owing to ongoing pathophysiological changes between the diseased and normal skin. This could be because of the nature of the inflammatory skin disease. In severe cases, psoriasis is often unstable and is composed of variable lesions, including borderline erythema, thin fine scaly skin-colored to erythematous papules, erythematous thick plaques, and thick plaques with silver-white scales. This may also be one of the main causes of discordance between dermatologists when evaluating the area of involvement. When evaluating a large image of a specific anatomical region, such as the trunk or extremities, these lesions all together in an individual image become truly complicated for machine learning. The excellent correlation of the estimated percentage of BSA involved between this U-net model and the dermatologist guides its promising use in clinical applications. We also proposed that, when developing a method for evaluating clinical applicability, the percentage of involvement, in addition to common parameters such as JI and DSC, be considered.

## 5. Conclusion

The area percentage of involvement is a crucial component of the calculation during systemic skin disease severity evaluation. Assessment is important during the treatment response evaluation. It is difficult for patients or physicians to accurately estimate the area of involvement by visual examination. Herein, the proposed methods with the U-net model are adopted to develop an efficient way to yield the result of the ratio of psoriasis-to-total skin as a percentage of involvement and to estimate the involved BSA, which shows a promising result.

The developed U-net model achieved dermatologist-level performance in estimating the BSA ratio for psoriasis. More data collection and benefits with respect to clinical decision-making should be performed in future studies.

## Figures and Tables

**Figure 1:** U-net architecture.

**Figure 2:** Performance for training and validation datasets.

**Figure 3:** Simulation results of the lowest residual percentage on different scales.

**Figure 4:** Images with three largest residual percentages.

**Figure 5:** Psoriasis area estimation for ground truth and test images.

**Figure 6:** Correlation scatterplots for U-net and dermatologist's segmentations.

**Figure 7:** Bland-Altman plots.

**Table 1:** Architectural details of the U-net.

# of layer	Layers in encoding path	Filter size	Output shape
Contraction path			
*L*_1_	Input		(512 × 512 × 3)
*L*_2_	Conv-1	3 × 3	(512 × 512 × 64)
*L*_3_	**Conv-2**	3 × 3	(512 × 512 × 64)
*L*_4_	Maxpool-1	2 × 2	(256 × 256 × 64)
*L*_5_	Conv-3	3 × 3	(256 × 256 × 128)
*L*_6_	**Conv-4**	3 × 3	(256 × 256 × 128)
*L*_7_	Maxpool-2	2 × 2	(128 × 128 × 128)
*L*_8_	Conv-5	3 × 3	(128 × 128 × 256)
*L*_9_	**Conv-6**	3 × 3	(128 × 128 × 256)
*L*_10_	Maxpool-3	2 × 2	(64 × 64 × 256)
*L*_11_	Conv-7	3 × 3	(64 × 64 × 512)
*L*_12_	**Conv-8**	3 × 3	(64 × 64 × 512)
*L*_13_	Maxpool-4	2 × 2	(32 × 32 × 512)
Expansion path			
*L*_14_	Conv-9	3 × 3	(32 × 32 × 1024)
*L*_15_	Conv-10	3 × 3	(32 × 32 × 1024)
*L*_16_	Upsampling-1	3 × 3	(64 × 64 × 1024)
*L*_17_	**Conv-11**	3 × 3	(64 × 64 × 512)
*L*_18_	Cat-1		(64 × 64 × 1024)
*L*_19_	Conv-12	3 × 3	(64 × 64 × 512)
*L*_20_	Conv-13	3 × 3	(64 × 64 × 512)
*L*_21_	Upsampling-2	3 × 3	(128 × 128 × 512)
*L*_22_	**Conv-14**	3 × 3	(128 × 128 × 256)
*L*_23_	Cat-2		(128 × 128 × 512)
*L*_24_	Conv-15	3 × 3	(128 × 128 × 256)
*L*_25_	Conv-16	3 × 3	(128 × 128 × 256)
*L*_26_	Upsampling-3	3 × 3	(256 × 256 × 256)
*L*_27_	**Conv-17**	3 × 3	(256 × 256 × 128)
*L*_28_	Cat-3		(256 × 256 × 256)
*L*_29_	Conv-18	3 × 3	(256 × 256 × 128)
*L*_30_	Conv-19	3 × 3	(256 × 256 × 128)
*L*_31_	Upsampling-4	3 × 3	(512 × 512 × 128)
*L*_32_	**Conv-20**	3 × 3	(512 × 512 × 64)
*L*_33_	Cat-4	3 × 3	(512 × 512 × 128)
*L*_34_	Conv-21	3 × 3	(512 × 512 × 64)
*L*_35_	Conv-22	3 × 3	(512 × 512 × 64)
*L*_36_	Conv-23	3 × 3	(512 × 512 × 32)
*L*_37_	Output	1 × 1	(512 × 512 × 3)

Conv = convolution; Maxpool = max-pooling; Upsampling = upsampling; Cat = concatenation.

**Table 2:** Description of the dataset.

Number of images by anatomical regions	Training	Validation	Testing	Total
Extremities	106	26	38	170
Trunk	59	15	11	85
Number of total images	165	41	49	255

**Table 3:** Partition of dataset.

Training dataset	Training patches	Validation patches	Testing images
Number of patches	7809	2048	×
Number of images	×	×	49

**Table 4:** Performance of testing datasets.

	ACC	Psoriasis			
		JI	DSC	SE	SP
Count	49	47	47	47	49
Mean	**0.976**	**0.536**	**0.655**	**0.657**	**0.988**
Std	**0.046**	0.267	0.256	0.227	0.033
Min	0.729	0.008	0.016	0.128	0.768
Q1	0.980	0.347	0.514	0.498	0.987
Q2	0.992	0.520	0.684	0.658	0.996
Q3	0.996	0.782	0.878	0.873	0.999
Max	0.999	0.958	0.979	0.983	1.000

**Table 5:** Performance indices with the smallest residual percentage.

	ACC	JI	DSC	SE	SP
Large scale	0.997	0.829	0.907	0.886	0.999
Small scale	0.969	0.869	0.93	0.921	0.982

**Table 6:** Residual percentage with test images.

	Residual percentage
Count	49
Mean	0.033
Std	0.076
Min	0.000
Q1	0.002
Q2	0.007
Q3	0.016
Max	0.398

**Table 7:** Parameters and file size for the proposed U-net, R2U-net, attention U-net, and attention R2U-net models.

	Proposed U-net	R2U-net	Attention U-net	Attention R2U-net
Parameters of model	31,035,971	32,086,440	31,902,759	32,261,767
Model file size	355 Mbytes	367 Mbytes	365 Mbytes	369 Mbytes

**Table 8:** Performances of testing datasets for the proposed U-net, R2U-net, attention U-net, and attention R2U-net models.

	Proposed U-net	R2U-net	Attention U-net	Attention R2U-net
Accuracy	0.976 (0.046)^∗^	0.967 (0.082)	0.960 (0.095)	0.969 (0.073)
JI	0.536 (0.267)	0.511 (0.244)	0.471 (0.230)	0.512 (0.258)
DSC	0.655 (0.256)	0.640 (0.233)	0.607 (0.223)	0.636 (0.247)
Sensitivity	0.657 (0.227)	0.550 (0.241)	0.523 (0.238)	0.599 (0.236)
Specificity	0.988 (0.033)	0.998 (0.003)	0.997 (0.004)	0.995 (0.006)

*m* (*s*)^∗^, *m* is the mean value, and *s* is the standard deviation.

**Table 9:** Residual percentage with test images for the proposed U-net, R2U-net, attention U-net, and attention R2U-net models.

	Proposed U-net	R2U-net	Attention U-net	Attention R2U-net
Count	49	49	49	49
Mean	0.033	0.070	0.094	0.067
Std	0.076	0.148	0.187	0.152
Min	0.000	0.000	0.000	0.000
Q1	0.002	0.004	0.004	0.003
Q2	0.007	0.010	0.008	0.009
Q3	0.016	0.054	0.079	0.029
Max	0.398	0.722	0.799	0.658

## Data Availability

The data used to support the findings of this study consisted of skin lesion images obtained from clinical records, and have not been made available to be publicly shared without approval from the institutional review board of the E-DA Hospital.
